# A Novel Formula Comprising Wolfberry, Figs, White Lentils, Raspberries, and Maca (WFWRM) Induced Antifatigue Effects in a Forced Exercise Mouse Model

**DOI:** 10.1155/2022/3784580

**Published:** 2022-03-24

**Authors:** Caixia Yang, Jingyan Yang, Li Tan, Pan Tang, Ting Pen, Tinghui Gao, Sijing Liu, Jinlin Guo

**Affiliations:** ^1^Key Laboratory of Characteristic Chinese Medicine Resources in Southwest China, College of Pharmacy, Chengdu University of Traditional Chinese Medicine, Chengdu 611137, China; ^2^College of Medical Technology, Chengdu University of Traditional Chinese Medicine, Chengdu 611137, China

## Abstract

Long-term body fatigue poses a threat to human health. To explore novel sources of antifatigue medicine and food, we developed a novel formula composed of wolfberry, figs, white lentils, raspberries, and maca (WFWRM) according to the theory of traditional Chinese medicine. In this study, we explored whether the administration of the WFWRM relieves fatigue. Thirty male Kunming mice were divided into three groups, which received either intragastric administration of saline, vitamin C (100 mg/kg), or WFWRM (1.00 g/kg) every day. After 30 days of treatment, all mice exhaustively performed weight-bearing swimming. Another ten mice that did not perform swimming were treated with saline for 30 days and used as sedentary control. The antifatigue effect and biochemical oxidation phenomena were assessed in the exercise-exhausted model and sedentary controls. The histopathological changes in the liver and kidney tissues of mice were observed by performing hematoxylin-eosin (HE) staining. After 30 days of oral administration, the liver and kidney tissues of mice were healthy and show no pathological changes. Compared to the fatigue model group, WFWRM significantly increased the rota-rod time of the mice. Also, the concentrations of lactic acid (LA), blood urea nitrogen (BUN), creatine kinase (CK), and lactate dehydrogenase (LDH) in the WFWRM group significantly reduced. On the contrary, the levels of hepatic glycogen (LG), muscle glycogen (MG), and serum glucose (GLU) increased in the WFWRM group. Besides, WFWRM markedly reduced the levels of malondialdehyde (MDA) but increased the levels of glutathione peroxidase (GSH-PX) and superoxide dismutase (SOD). Pearson correlation analysis indicated that the concentrations of the sources of energy (LG, MG, and GLU) significantly correlated with those of metabolites (BLA, BUN, CK, and LDH) and antioxidant levels (SOD, GSH-PX, and MDA). Overall, our results suggested that the supplementation of WFWRM could improve exercise capacity and relieve fatigue probably by normalizing energy metabolism and attenuating oxidation.

## 1. Introduction

Fatigue refers to the inability of the body to maintain its function at a specific level or to achieve the predetermined exercise intensity [1]. Based on the development process of fatigue, it can be divided into acute, chronic, and excessive fatigue [2]. Acute fatigue can be recovered to normal after a long rest, but chronic and excessive fatigue are suboptimal health states that cannot be recovered only by resting and usually lead to aging, metabolic disorder, depression, and cancer [2]. These symptoms can seriously affect the learning efficiency, quality of life, and work progress of people. Some chemical drugs, such as modafinil, amphetamine, and methylphenidate are available to relieve fatigue, but the side effects of those chemical drugs, including mental disorders, drowsiness, and addiction, were commonly reported and might limit their application [3–5]. Therefore, additional strategies that alleviate fatigue are required.

The pathogenesis of fatigue remains unclear, although increasing evidence suggests that it is mainly related to energy exhaustion and accumulation of metabolites and free radicals [6, 7]. Carbohydrates in the body are mainly in the form of hepatic glycogen (LG) and muscle glycogen (MG) in tissue cells and serum glucose (GLU) in the blood [8, 9]. During exercise, these energy sources are exhausted, leading to fatigue. The concentrations of LG, MG, and GLU are, therefore, used to evaluate fatigue. Additionally, a large amount of urea nitrogen (BUN) is generated when protein metabolizes to produce energy. After exercise, the increase in metabolites, such as BUN and lactic acid (LA), can decrease the vitality of muscle cells, affect enzyme activity (LDH and CK), and reduce energy production, resulting in fatigue [10, 11]. Free radicals are also considered the main factor that contributes to fatigue. The accumulation of free radicals can cause lipid peroxidation of the mitochondrial membrane, inhibit cell respiration, induce the oxidation of energy substances and lead to fatigue [12]. Glutathione peroxidase (GSH-PX) and superoxide dismutase (SOD) are important antioxidant enzymes, which can scavenge free radicals and reduce the production of malondialdehyde (MDA) to resist exercise-induced oxidative damage and relieve fatigue [13].

It is reported that several plant extracts or Chinese traditional medicines containing alkaloids, flavonoids, and polyphenols not only reduce fatigue but also have the advantage of having fewer side effects [14]. Therefore, based on the theory of Chinese traditional medicine, we developed a novel formula composed of wolfberry, figs, white lentils, raspberries, and maca (WFWRM) and hypothesized that it would have an antifatigue effect. Several studies demonstrated the high antioxidant activity of wolfberry; it could scavenge free radicals in high-fat-fed rats and inhibit the peroxidation of low-density lipoprotein (LDL) [15, 16]. Meanwhile, it has been reported that maca contains flavonoids and alkaloids, is neuroprotective, and improves swimming endurance capacity in ICR mice [17]. Previous studies demonstrated that white lentils, figs, and raspberries have antioxidant effects, but there are only a few reports of their antifatigue activity [18–20]. In the current study, we set out to explore the efficacy of WFWRM to relieve fatigue, using a well-established weight-bearing swimming mouse model.

## 2. Materials and Methods

### 2.1. Chemicals, Reagents, and Materials

Bicinchoninic acid (BCA) protein determination kits were provided by Boster Biological Engineering Co. Ltd (Wuhan, China). Lactic acid (LA), blood urea nitrogen (BUN), muscle glycogen (MG), liver glycogen (LG), malondialdehyde (MDA), superoxide dismutase (SOD), and glutathione peroxidase (GSH-PX) determination kits were purchased from Enzyme Link Biotechnology Co. Ltd (Shanghai, China). Creatine kinase (CK), lactate dehydrogenase (LDH), and glucose (GLU) determination kits were purchased from Mindray Biological Technology Co. Ltd (Shenzhen, China).

### 2.2. Preparation of WFWRM and Compositional Analysis

The formulation of WFWRM is presented in Table 1. The Chinese medicinal herbs were made into tablets by Shanghai Tianyuan Plant Products Co. Ltd (Shanghai, China). The company mixed the powders of wolfberry, fig, white lentils, raspberry, and maca and boiled them in water (material-liquid ratio = 1 : 10) for 2 hours to obtain the extract. Then, the aqueous extract was spray dried and tabletted to obtain WFWRM. In this study, we dissolved WFWRM in normal saline for gavage. Moreover, the phytochemical characterization of WFWRM was performed on an UPLC-Q-Orbitrap High Resolution Mass Spectrometer (Thermo Fisher Scientific Company, USA) using both positive and negative modes. The WFWRM powder (1.09 g) was added to 100 mL methanol and was then extracted for 60 min in a water bath at 60°C. The extract was centrifuged at 4,000*g* for 10 min, and the supernatant was filtered with a 0.22 *μ*m nylon filter membrane. The WFWRM extract was separated using a Thermo Scientific AccucoreTM C18 column (2.6 *μ*m, 3 mm × 100 mm). The temperature of the column was 40°C, and the sample injection volume was 5 *μ*L. The eluents were 0.1% formic acid (A) and acetonitrile (B). The flow rate was 0.2 mL/min, and the gradient program started at 95% A and held at 95% A for 1 min, decreased to 5% A for 20 min, held at 5% A for 1 min, increased to 95% A for 0.1 min, and held at 95% A for 0.9 min. The parameters of mass spectrometry were set as follows: scanning range, 100–1500 m/z; spray voltage, 3 kV; sheath gas volume flow, 35 arb; auxiliary gas volume flow, 10 arb; auxiliary device temperature, 250°C; and the temperature of the ion transfer tube, 300°C.

### 2.3. Animals and Experimental Design

Healthy male Kunming mice (specific pathogen free, SPF) used in this study were supplied by the Dashuo Laboratory Animal Co. Ltd. (Chengdu, China). All experiments were performed according to the guidelines by the Animal Research Committee of the Chengdu University of Traditional Chinese Medicine. They were 5 weeks old and their body weights were 22 ± 3 g, and they were kept in a temperature (22 ± 2°C) and humidity (55 ± 15%) controlled room at a 12-hour light/dark cycle. All mice were allowed free access to distilled water and a rodent chow diet throughout the experimental period. After adaptive feeding for one week, 40 mice were randomly divided into 4 different groups (*n* = 10): (1) the sedentary control group (CON) mice were treated with saline daily for 30 days without weight-bearing swimming; (2) the model group (MOD) mice were treated with saline by oral gavage daily for 30 days and then were exhaustively exercised through weight-bearing swimming; (3) the vitamin C group (VC) mice were daily treated with vitamin C (100 mg/kg) by oral gavage daily for 30 days and then exhaustively exercised through weight-bearing swimming; and (4) the WFWRM treatment group (WFWRM) mice were treated with WFWRM (1.00 g/kg) by intragastric administration (0.2 mL/10 g) daily for 30 days and then exhaustively exercised through weight-bearing swimming. In order to evaluate the safety of WFWRM, another 9 mice were also randomly divided into 3 different groups (*n* = 3): the CON group, the VC group, and the WFWRM treatment group. They were daily gavaged with saline, vitamin C (100 mg/kg), and WFWRM (1.00 g/kg) for 30 days without the rota-rod test and the swimming exhaustion experiment. The doses were decided based on the recommended human dose [21]. The general food intake was monitored every day, and the body weight was recorded every five days.

### 2.4. Rota-Rod Test and Histopathological Analysis

After treatment for 30 min on the 28^th^ day, mice from each group were trained on a Fatigue Rotary Rod Apparatus ZB-200 (Chengdu Taimeng Science Technology Co. Ltd, Chengdu, China) at 15 rpm [22]. In the formal test, mice were placed on the rota-rod at 15 rpm, until they were exhausted and dropped from the rod, and the total running time was measured. Three mice from each group were not subjected to the rota-rod test or the swimming exhaustion experiment, and the internal organs, such as liver and kidney, and skeletal muscles of the hind legs were collected. The liver and kidney tissues were fixed in 4% paraformaldehyde, embedded in paraffin, and cut into 4 *μ*m thick sections. The sections were stained with HE and observed using a light microscope (Olympus, Tokyo, Japan) to evaluate the pathological changes.

### 2.5. Weight-Loaded Forced Swimming and Sample Collection

The weight-loaded forced swimming test (WFST) was carried out in a swimming pool (40 × 46 × 63 cm) with 30 cm deep water, maintained at 25 ± 1°C. On the 30^th^ day, each mouse was loaded with a lead block (4% of the body weight) and was given a swimming exercise for 30 min. If a mouse was floating during the experiment, it would be forced to swim by stirring the water with a glass rod [22]. After 30 minutes, all mice were removed from the water and dried using a towel. Mice were sacrificed, and the serum, liver, and skeletal muscles of the hind legs were collected. All samples were stored at −80°C until use.

### 2.6. Determination of Biochemical Parameters in the Serum, Liver, and Muscles

Serum LA, serum BUN, muscle MG, and liver (MDA, SOD, GSH-PX, and LG) parameters were measured using the ELISA kits, in accordance with the manufacturer's instructions. The LDH, GLU, and CK levels were determined using the Mindray BS-200 automatic biochemical analyzer (Mindray Biological Technology Co. Ltd, Shenzhen, China) using the diagnostic kits, in accordance with the manufacturer's instructions.

### 2.7. Data Analysis

Statistical analysis was performed using GraphPad Prism 9 (San Diego, CA, USA) and SPSS 22.0 software (IBM, USA). All data were expressed as mean ± SD. One-way ANOVA with a LSD-*t* or Dunnett multiple comparison test was used for comparison among three groups. The correlation between energy metabolites and antioxidant-related traits was evaluated using Pearson correlation analysis. *P* < 0.05 was considered statistically significant difference.

## 3. Results and Discussion

### 3.1. Chemical Compounds in WFWRM

In this study, we analyzed WFWRM using data-dependent UPLC-Q-TOF-MS, using both positive and negative polarity modes. After data comparison using the PubChem, ChemSpider, mzCloud, and mzVault databases and corresponding literature, twenty-seven constituents of WFWRM were identified, which are presented in Table 2. We found that the components of WFWRM were amino acids and metabolites (DL-arginine, 2-hydroxyphenylalanine, L-phenylalanine, and indole-3-acrylic acid), flavonoids (formononetin, (+)-ar-turmerone, isoliquiritigenin, butein, kaempferol, catechin, trifolin, and rutin), polyphenols (gallic acid and curcumin), alkaloids (DL-stachydrine, caffeine, and trigonelline), fatty acids (9-Oxo-ODE, 12,13-DiHOME, 9S,13R-12-oxophytodienoic acid and 9-HpODE), terpenoids (18-*β*-glycyrrhetinic acid, zerumbone, (−)-caryophyllene oxide and (±)-abscisic acid), and others (1-linoleoyl glycerol and palmitoylethanolamide). These chemical compounds may be the material basis of WFWRM to resist fatigue. A previous study indicated that patients with amino acid deficiency may develop dysfunctions of the pain-inhibitory mechanisms together with fatigue [23]. Consistent with this conclusion, Chen et al. recently showed that L-arginine supplementation could minimize skeletal muscle damage and reduce the accumulation of free radicals to decrease the occurrence of fatigue in rats [24]. Moreover, L-phenylalanine is a potential lipophilic antioxidant. Physalis pubescens *L* contains L-phenylalanine and other metabolites that relieve fatigue in rats by ameliorating the disturbances in amino acids and energy metabolism, alleviating the oxidative stress due to the reactive oxygen species [25]. Besides, 2-hydroxyphenylalanine is an isomeric tyrosine derived from L-phenylalanine and can participate in amino acid metabolism to provide energy to the body [26]. Flavonoids polyphenols, which are promising natural plant antioxidants, resist fatigue by scavenging free radicals and reducing the transfer speed of the auto-oxidation chain reaction [27]. For instance, there are reports suggesting that the catechin of grape seeds, rutin, curcumin, and kaempferol were able to extend the swimming time of weighted mice before exhausting by reducing the accumulation of free radicals, increasing the activity of antioxidant enzymes (GSH-PX, CAT, and SOD), and decreasing the production of metabolites (BUN and BLA) [27, 28]. The application of alkaloids to relieve fatigue is increasingly being considered. Caffeine and trigonelline are hallmark plant alkaloids in coffee that increase athletic ability [29]. A study has shown that male participants who consumed low caffeine showed better fatigue resistance of the knee flexors, compared to those in the control group [30]. Similarly, trigonelline has been reported to decrease apoptosis and restore the MDA content in unilaterally 6-OHDA-lesioned rats [31]. Moreover, trigonelline could reduce oxidative stress and insulin resistance to maintain normal blood glucose in type-2 diabetes mellitus rats [32]. Fatty acids are also reported to have the effect of resisting cancer-related fatigue [33]. For instance, 9-oxo-ODE could strongly activate the antioxidant response element to lessen the damage caused by oxidative stress [34]. Moreover, 12,13-DiHOME increased fatty acid uptake and oxidation in skeletal muscles of mice, which was able to reduce the production of free fatty acids and prevent tryptophan in the plasma from entering the brain to resist fatigue [35]. In addition, peripheral inflammation and immune activation Meanwhile, palmitoylethanolamide is a fatty acid derivative that can antifatigue through inhibiting inflammation [36]. Notably, it has been reported that the treatment of Baoyuan Jiedu decoction involving indole-3-acrylic acid, isoliquiritigenin, formononetin, 18-*β*-glycyrrhetinic acid, and 9S,13R-12-oxophytodienoic acid prevented prominent myotube atrophy and regulated mitochondrial production [37]. Indeed, mitochondria and muscles are damaged with fatigue [38]. Therefore, the protection of muscles and mitochondria may relieve fatigue to a greater extent. Although no studies have shown that DL-stachydrine, (+)-ar-turmerone, gallic acid, butein, trifolin, zerumbone, 1-linoleoyl glycerol, (−)-caryophyllene oxide, and (±)-abscisic acid can relieve fatigue. However, studies have shown that they exhibit antioxidant activities towards oxidative stress and antioxidants are essential for relieving fatigue [39–47]. Since, WFWRM contains these components, we speculated that it has an antifatigue effect.

### 3.2. WFWRM Increased the Rota-Rod Time

Exercise endurance is a direct indicator of fatigue and the rota-rod time has been used to evaluate the antifatigue effect in several studies [48, 49]. In this study, we determined the rota-rod time after 30 days of WFWRM supplementation. As shown in Figure 1(a), WFWRM markedly increased the rota-rod time by 147.07% compared to the model group (*P* < 0.001). We used vitamin C as a positive control drug, which is usually used for resisting fatigue and could reduce oxidative damage due to exercise [50]. The rota-rod time of mice in the vitamin C treatment group was 41.75% higher than that in the model group (*P* < 0.0001). Surprisingly, WFWRM had a better effect on the rota-rod time compared to vitamin C. Therefore, it is reasonable to assume that WFWRM is a promising agent for relieving fatigue. Moreover, the food intake (Figure 1(b)) and body weight (Figure 1(c)) were not affected by WFWRM (*P* > 0.05). We also found that there were no significant histological changes in the livers and kidneys of mice across the different groups (Figure 2), suggesting that WFWRM is a safe and promising approach to relieve fatigue. These results indicated that WFWRM could significantly enhance the exercise capacity of mice without any damage.

### 3.3. WFWRM Increased Serum Glucose Levels and Liver and Muscle Glycogen Levels in Exhaustive Mice

GLU is an important component of the body and an important source of energy for various tissues and organs [51]. In addition to maintaining optimum GLU levels, the excess sugar ingested by the body is stored in the form of LG and MG [8]. During vigorous exercise, if GLU is not sufficient, LG is broken down into GLU [9]. During prolonged and strenuous exercise, MG can also be converted into LG to supply energy [52]. Increased storage of GLU, LG, and MG could enhance endurance and exercise capacity. Therefore, the serum GLU, LG, and MG levels can reflect the degree of fatigue. In this study, we found that the serum GLU (*P* < 0.0001), LG (*P* < 0.01), and MG (*P* < 0.01) levels of WFWRM-treated mice were significantly increased by 75.1%, 43.5%, and 36.1%, respectively (Figure 3). These results suggested that the improvement in the antifatigue activity of WFWRM may be related to the homeostatic ability of blood glucose.

### 3.4. WFWRM Decreased Serum BUN, LA, CK, and LDH Levels

As the intensity of exercise increases, carbohydrates and fats may not meet the energy needs. Proteins, thus, will be consumed and produce a large number of nitrogen-containing compounds and *α*-keto acids [53]. The former is converted into urea and excreted via urine, while the latter is used as a raw material for the synthesis of glucose [54, 55]. Therefore, BUN, the final by-product of protein metabolism, can be used to evaluate protein mobilization and fatigue. In the present study, WFWRM reduced the production of BUN by 40.9% compared to the model group (Figure 4(a), *P* < 0.0001). This suggests that WFWRM reduced the consumption of protein in mice during exercise and showed antifatigue activity. During vigorous exercises in a short period, the oxygen-carrying capacity of the body becomes insufficient, resulting in anaerobic respiration by the muscle cells [56]. Anaerobic glycolysis produces LA while supplying energy, which could damage organs and lead to fatigue by lowering pH [57]. CK is an important enzyme responsible for muscle contraction and ATP regeneration [58]. LDH exists in almost all organs and tissues but its content in the blood is very low. However, when the cells are destroyed, the blood LDH levels rise [59, 60]. Therefore, the cytosolic enzymes, LA, CK, and LDH can be used to evaluate the extent of muscle damage and the degree of fatigue. The more vigorous and longer the exercise, the higher the levels of LA, CK, and LDH. In this study, the content of LA, CK, and LDH increased significantly in the MOD as compared to the CON (Figure 4(b), *P* < 0.0001). Compared to the MOD, the levels of LA, CK, and LDH decreased by 34.0%, 43.5%, and 33.5% in WFWRM, respectively (Figures 3(b)–3(d), *P* < 0.0001). These findings suggested that WFWRM may reduce the damage to the muscle cells in mice, which may be related to its antifatigue activity.

### 3.5. WFWRM Increased Antioxidant Activity and Decreased the MDA Level

It has been reported that oxidative stress is closely related to fatigue even though the mechanism is still unclear. SOD is a catalytic enzyme that converts oxygen free radicals into H_2_O_2_ [61]. H_2_O_2_ is decomposed into O_2_ and H_2_O under the catalysis of GSH-PX and CAT (catalase) [62]. When the content of SOD and GSH-PX in the body is low, free radicals obtain electrons from the cell membrane, damage the mitochondrial membrane, and cause lipid peroxidation [63]. Moreover, MDA is the end product of lipid peroxidation. Previous studies indicated that mice gavaged with polysaccharides from *Lepidium meyenii* Walp. (maca) or *Lycium ruthenicum* show inceased GSH-PX and SOD levels and decreased the MDA levels [64, 65]. In our study, exhaustive exercise did not affect the hepatic concentration of GSH-PX and SOD, but significantly increased the hepatic MDA levels (*P* < 0.05). The content of GSH-PX and SOD increased by 49.8% and 59.4%, respectively, while that of MDA decreased by 24.4% after WFWRM treatment (*P* < 0.0001, Figure 5). Our results indicated that the WFWRM supplementation attenuated the oxidative stress and might help restore the oxidant-antioxidant balance.

### 3.6. Pearson Correlation Analysis among the Different Indicators

The Pearson correlation analysis is used to analyze the direction and degree of linear correlation between two variables [66]. In this study, we used Pearson correlation analysis to evaluate the correlation between the different indicators. As shown in Figure 6, all possible pairs of LDH, BUN, LA, and CK showed a significant positive correlation (*P* < 0.001). There was no significant correlation between LG, MG, and GLU (*P* > 0.05). SOD and GSH-PX were positively correlated (*P* > 0.001). However, SOD and MDA were negatively correlated (*P* < 0.05). Overall, these results indicated that WFWRM administration could effectively reduce the accumulation of metabolites while increasing the activity of antioxidant enzymes to maintain optimum blood glucose levels even after weight-bearing swimming.

## 4. Conclusion

Gavaged with the novel formula comprising wolfberry, figs, white lentils, raspberries, and maca, the mice showed increased exercise ability as assessed by the rota-rod test and accelerated the metabolism of lactic acid and urea nitrogen to relieve fatigue. Also, the novel formula decreased the activity of creatine kinase and lactate dehydrogenase to reduce the occurrence of fatigue. Moreover, the novel formula also resisted fatigue by increasing the activity of antioxidant enzymes and reducing malondialdehyde production to reduce oxidative stress. In addition, we found that the main components of the novel formula were amino acids, alkaloids, and fatty acids. These chemical compounds may contribute to its antifatigue activity. In short, the novel formula showed a significant antifatigue effect and had the potential to develop into an antifatigue supplement (Figure 7).

## Figures and Tables

**Figure 1:** Rota-rod time, food intake, and body weight in different groups. Normal mice or exhaustive exercised mice were treated with saline, vitamin C (100 mg/kg), and WFWRM (1.00 g/kg) for 30 days by oral gavage. (a) Rota-rod time. (b) Food intake. (c) Body weight. Data were represented as mean ± SD. All experiments were performed three times. The differences of data among the three groups were analyzed by one-way ANOVA with the LSD-t multiple comparisons test. ^####^*P* < 0.0001, compared with the model group. CON, control group. MOD, model group. VC, vitamin C group. WFWRM, the novel formula group (*n* = 10).

**Figure 2:** WFWRM did not affect histopathology of livers and kidneys (hematoxylin-eosin staining, 100×). Normal mice or exhaustive exercised mice were treated with saline, vitamin C (100 mg/kg), and WFWRM (1.00 g/kg) for 30 days by oral gavage. (a–c) Livers and (d–f) kidneys were collected and stained with hematoxylin-eosin staining. Histopathology changes in the liver and kidney were observed and photographed under a microscope (magnification, 100x). CON, control group. VC, vitamin C group. WFWRM, the novel formula group.

**Figure 3:** Effects of the WFWRM on antifatigue glycogen and glucose content indicators. Normal mice or exhaustive exercised mice were treated with saline, vitamin C (100 mg/kg), and WFWRM (1.00 g/kg) for 30 days by oral gavage. (a) GLU, (b) LG, and (c) MG content in the serum. All experiments were performed three times. Data were expressed as mean ± SD. One-way ANOVA with the LSD-(t) or Dunnett multiple comparisons test was used for comparison between the three groups, ^*∗∗*^*P* < 0.01 and ^*∗∗∗∗*^*P* < 0.0001, compared with MOD. CON, control group. MOD, model group. VC, vitamin C group. WFWRM, the novel formula group (*n* = 10).

**Figure 4:** Effects of the WFWRM on anti-fatigue biochemical indicators. Normal mice or exhaustive exercised mice were treated with saline, vitamin C (100 mg/kg), and WFWRM (1.00 g/kg) for 30 days by oral gavage. (a) BUN, (b) LDH, (c) LA, and (d) CK concentrations of each group in the serum. All experiments were performed three times. Data were expressed as mean ± SD. One-way ANOVA with the LSD-(t) or Dunnett multiple comparisons test was used for comparison between the three groups, ^*∗∗*^*P* < 0.01 and ^*∗∗∗∗*^*P* < 0.0001, compared with MOD. ^####^*P* < 0.0001, compared with CON. CON, control group. MOD, model group. VC, vitamin C group. WFWRM, the novel formula group (*n* = 10).

**Figure 5:** Effect of the WFWRM on antifatigue oxidative indicators. Normal mice or exhaustive exercised mice were treated with saline, vitamin C (100 mg/kg), and WFWRM (1.00 g/kg) for 30 days by oral gavage. (a) GSH-PX, (b) SOD, and (c) MDA content in the liver. All experiments were performed three times. Data were expressed as mean ± SD. One-way ANOVA with the LSD-(t) multiple comparisons test was used for comparison between the three groups. ^*∗*^*P* < 0.05 and ^*∗∗∗∗*^*P* < 0.0001, compared with MOD. ^#^*P* < 0.05, compared with CON. CON, control group. MOD, model group. VC, vitamin c group. WFWRM, the novel formula group (*n* = 10).

**Figure 6:** Correlations between carbohydrate metabolism and metabolite- and oxidative stress-related parameters. Pearson correlation analysis was calculated for all experimentally determined parameters in this study. The R values are presented by gradient colors, where red and blue indicate positive and negative correlations, respectively. The asterisks ^*∗*^, ^*∗∗*^, and ^*∗∗∗*^ indicated *P* < 0.05, *P* < 0.01, and *P* < 0.001, respectively.

**Figure 7:** Illustration of the antifatigue effect of WFWRM through regulating antifatigue-related biochemical indicators. The WFWRM inhibited mitochondrial lipid peroxidation by increasing antioxidant enzymes (SOD and GSH-PX) and reducing the level of MDA. The downregulation of LDH and LA was responsible for the restraint of antifatigue by restraining the lactic acid shuttle mechanism. The upregulation of storing or mobilizing MG and LG could increase the concentrations of GLU to provide energy directly to antifatigue in the body. The WFWRM could relieve fatigue caused by muscle damage by decreasing the production of CK, reducing protein consumption, and accelerating the metabolism of BUN.

**Table 1:** The formulations of WFWRM.

Common name	Herb name	Family name	Part used	Amount used (g/d)
Maca	*Lepidium meyenii* Walp	Brassicaceae	Dry roots and rhizomes	15
Raspberry	*Rubus chingii* Hu	Rosaceae	Dry fruit	10
Fig	*Ficus carica* Linn	Moraceae	Dry ripe fruit	20
Wolfberry	*Lycium barbarum* L	Solanaceae	Dry ripe fruit	10
White lentil	*Lablab semen* Album	Leguminosae	Dry ripe fruit	10

**Table 2:** Compounds from WFWRM identified by UPLC-ESI-MS.

Name	Molecular formula	Molecular weight	Rt (min)	Area (Max)	M/Z	Fragments
DL-Arginine	C_6_H_14_N_4_O_2_	174.1117	1.248	4.40 × 10^9^	175.1189	116.0708, 70.0657
18-*β*-Glycyrrhetinic acid	C_30_H_46_O_4_	470.3395	10.643	1.60 × 10^9^	471.3467	453.3362, 189.1636
Indole-3-acrylic acid	C_11_H_9_NO_2_	187.0635	4.169	1.26 × 10^9^	188.0705	170.0560, 146.0506
DL-Stachydrine	C_7_H_13_NO_2_	143.0947	1.328	1.17 × 10^9^	144.1019	98.0604, 84.0813
Formononetin	C_16_H_12_O_4_	268.0735	11.015	9.58 × 10^8^	269.0806	237.0543, 118.0415
(+)-ar-Turmerone	C_15_H_20_O	216.1515	16.852	4.35 × 10^8^	217.1052	119.0857, 91.0547
Gallic acid	C_7_H_6_O_5_	170.0211	1.977	4.18 × 10^8^	169.0137	125.0236, 97.0286
Caffeine	C_8_H_10_N_4_O_2_	194.0806	4.967	3.87 × 10^8^	195.0876	138.0661, 110.0715
9-Oxo-ODE	C_18_H_30_O_3_	294.2196	10.355	3.66 × 10^8^	295.2262	277.2163, 99.0809
2-Hydroxyphenylalanine	C_9_H_11_NO_3_	181.074	1.674	3.46 × 10^8^	182.0811	165.0546, 147.0440, 136.0757
Trigonelline	C_7_H_7_NO_2_	137.0477	1.601	3.27 × 10^8^	138.0551	110.0678, 94.0655
Isoliquiritigenin	C_15_H_12_O_4_	256.0736	6.439	2.88 × 10^8^	257.0806	137.0233, 119.0493
Curcumin	C_21_H_20_O_6_	368.126	10.143	2.53 × 10^8^	369.1332	259.0967, 177.0546
Butein	C_15_H_12_O_5_	272.0686	7.809	1.97 × 10^8^	273.0755	137.0233, 91.0546
12 (13)-DiHOME	C_18_H_34_O_4_	314.2461	13.741	1.92 × 10^8^	313.2386	295.2275, 183.1385, 129.0913
9S,13R-12-Oxophytodienoic acid	C_18_H_28_O_3_	292.2037	15.893	1.60 × 10^8^	293.2092	275.2001, 79.0548
Kaempferol	C_15_H_10_O_6_	286.048	10.007	1.45 × 10^8^	287.0548	165.0182, 153.0182, 121.0286
Palmitoylethanolamide	C_18_H_37_NO_2_	299.2825	19.376	9.80 × 10^7^	300.3242	283.2629, 62.0607
Zerumbone	C_15_H_22_O	218.1672	13.727	8.72 × 10^7^	219.1742	135.0804, 107.0858, 67.0548
Catechin	C_15_H_14_O_6_	290.0794	4.834	8.59 × 10^7^	291.0858	165.0546, 139.0389, 123.0441
L-Phenylalanine	C_9_H_11_NO_2_	165.0791	2.194	5.44 × 10^7^	166.0859	142.9669, 120.0809, 103.0545
Trifolin	C_21_H_20_O_11_	448.1012	7.121	5.08 × 10^7^	449.1715	287.0547
1-Linoleoyl glycerol	C_21_H_38_O_4_	354.2769	16.42	4.14 × 10^7^	355.2835	337.2741, 263.2367
Rutin	C_27_H_30_O_16_	610.1542	6.374	2.73 × 10^7^	609.1462	300.0277, 271.0249
(−)-Caryophyllene oxide	C_15_H_24_O	220.1829	18.446	2.47 × 10^7^	221.1899	203.1794, 111.1171
9-HpODE	C_18_H_32_O_4_	312.2307	14.287	1.42 × 10^7^	311.2231	293.2124, 197.1180
(±)-Abscisic acid	C_15_H_20_O_4_	264.1364	8.784	7.28 × 10^6^	263.1291	219.1387, 204.1151, 136.0522

## Data Availability

The data used to support the findings of this study are included within the article.
